The article "Awareness and Utilization of Affordable Medicine Facility-Malaria among Caregivers of Under-Five Children in Ibadan North-West Local Government Area, Oyo State" was published in 2013. Journal: Malar Res Treat.

# Awareness and Utilization of Affordable Medicine Facility-Malaria among Caregivers of Under-Five Children in Ibadan North-West Local Government Area, Oyo State

**DOI:** 10.1155/2013/176096

**Published:** 2013-12-30

**Authors:** Ikeoluwapo O. Ajayi, Tolulope Soyannwo, Onoja M. Akpa

**Affiliations:** ^1^Department of Epidemiology and Medical Statistics, College of Medicine, University of Ibadan, Ibadan, Nigeria; ^2^Department of Preventive Medicine and Primary Care, University of Ibadan, Ibadan, Nigeria

## Abstract

*Introduction*. Distribution of Affordable Medicine Facility-malaria Artemisinin Combination Therapies (AMFm-ACTs) started in Nigeria in 2011, but its use at community level has not been documented. *Methods*. Four hundred seventy-eight caregivers whose under-five children had fever within two weeks prior to the survey were selected using cluster sampling technique. Information on sociodemographic characteristics, treatment seeking for malaria, and awareness and use of AMFm-ACTs was collected using an interviewer administered questionnaire. *Result*. More than half of the respondents (51.2%) bought AMFm-ACTs without prescription. Awareness of AMFm was low as only 9.1% has heard about the programme. Overall, 29.2% used AMFm-ACTs as their first line choice of antimalarial drug. On bivariate analysis age, group (25–34 years), public servants, respondents with tertiary education, respondents with high socioeconomic status, respondents with poor knowledge of symptoms of malaria, awareness of AMFm-ACTs, availability of AMFm-ACTs, and sources of drug were significantly associated with utilization of AMFm-ACTs (*P* < 0.05). Logistic regression demonstrated that only people who were aware of AMFM-ACTs predicted its use (AOR: 0.073; CI: 0.032–0.166; *P* < 0.001). *Conclusion*. Interventions which targeted at raising awareness of AMFm-ACTs among people at risk of malaria are advocated for implementation.

## 1. Background

High malaria morbidity and mortality have persisted because of failed transactions between those at risk of malaria infection and available effective antimalarial drugs and preventive measures [1]. Artemisinin-Based Combination Therapies (ACTs), the most effective drugs to treat *Plasmodium falciparum,* malaria were recommended by World Health Organization (WHO) in 2001 for malaria endemic countries following resistance to the cheap and the long used antimalarials such as chloroquine, sulfadoxine-pyrimethamine, and amodiaquine and the resultant increasing burden of malaria [2]. Since the introduction, distribution of ACT has been slow [2]. Nigeria adopted ACT in 2005 and like the situation in other endemic countries access to ACTs by most people at risk of malaria has been a challenge. The ACTs are not widely used because of their high price, unreliable public sector supply, limited availability in the private sector, and patient self-medication with less expensive monotherapies [3].

The article "Awareness and Utilization of Affordable Medicine Facility-Malaria among Caregivers of Under-Five Children in Ibadan North-West Local Government Area, Oyo State" was published in 2013. Journal: Malar Res Treat.

In response to the low ACT access and the threat of artemisinin resistance developing in malaria parasite, the Institute of Medicine released a report in 2004 recommending the creation of a global subsidy (by reducing the price of the drugs at the manufacturer level) and that ACTs be made available through both the public and private sectors at the same price as chloroquine and other common therapies [2]. According to the Institute, the subsidy is expected to expand access to ACTs, crowd out monotherapies, decrease resistance to ACTs, and therefore decrease the burden of malaria. This concept was later developed by the Roll Back Malaria Partnership into a global mechanism known as the Affordable Medicines Facility-malaria. Global Fund hosted the AMFm-ACTs subsidy project in 2009 [3].

Affordable Medicine Facility-malaria-ACTs distribution channels involve both the public and private sectors. The private sector was included because studies done previously indicated that the majority of patients in many malaria endemic countries seek treatment outside of the formal public sector, with a large proportion accessing treatment through the private sector instead. Private sector treatment sources vary considerably between and within countries, ranging from private hospitals and clinics to one-room drug shops, general stores, and medicine peddlers [4]. Studies revealed that patients seek malaria treatment in the private sector—because of long distance to, long waiting time at, and stock out of drugs in the public sector as well as shortage of skilled providers [5].

Nigeria was one of the countries selected for AMFm phase 1 distribution. Nigeria started the distribution of AMFm-ACTs in 2011 firstly in the private sector then later in public sector. Society for Family Health (SFH), through the Global Fund Malaria and Prepackaged Therapy (PPT) projects, is working to ensure broad access to ACTs in Nigeria. Through the Global Fund under the AMFm-ACT initiative, SFH is providing a subsidized form of artemether-Lumefantrine (AL) known as ACTm. These medicines are distributed through private health care providers including proprietary patent medicine vendors (PPMVs) (local drug shopkeepers) and community-based pharmacies. SFH works closely with the Federal Ministry of Health on technical matters, education, training, and coordinating policy formulation and research to move the nation forward on both prevention and treatment issues in her battle against malaria.

The article "Awareness and Utilization of Affordable Medicine Facility-Malaria among Caregivers of Under-Five Children in Ibadan North-West Local Government Area, Oyo State" was published in 2013. Journal: Malar Res Treat.

While some effort at studying the adherence of drug distributors to use of AMFm-ACTs has been documented, its use at the community level is yet to be studied. Information on awareness of AMFM-malaria and how it has affected its use is lacking. Several past studies have concentrated on provider's knowledge on the drug and availability of the drugs at facilities where they are distributed. Hence, this study aimed at determining awareness, utilization, and factors influencing utilization of AMFm-ACTs in communities in Ibadan North-West Local Government.

## 2. Methods

### 2.1. Study Area

The study was conducted in Ibadan North-West Local Government Area which is one of the eleven LGAs that constitute Ibadan metropolitan area. Ibadan is the capital of Oyo state, one of the 36 states of the Federal Republic of Nigeria. The state is centrally situated in the southwestern part of the country and is 128 km north-east of Lagos and 345 km south-west of Abuja, the federal capital territory. For administrative purposes the city is divided into 11 Local Government Areas (LGAs), five of which are urban. Ibadan North-West is one of the five urban LGAs. It has a population of 152,834 people based on 2006 census [6]. The inhabitants of Ibadan North-West LGA are mostly Yoruba while the main occupations of the people are trading and working in the public service. There are 11 political wards and 6 primary health centres (government owned) in the local government [7]. Treatment of malaria takes place in health facilities and at other healthcare providers' places such as private patent medicine shops (PPMVs), pharmacy shops and appointed community medicine distributors. However, home management of malaria using drugs bought from PPMVs and pharmacy is a common practice among caregivers in Nigeria including those in this study LGA.

### 2.2. Study Design and Population

#### 2.2.1. Study Design

This was a cross-sectional study and cluster sampling technique was used in selecting caregivers who participated in the study.

#### 2.2.2. Study Population

Women caregivers in their reproductive age (15–49 years) whose children had fever within two weeks prior to the survey were included in the study. It was estimated that a minimum sample size of 430 caregivers will be required to estimate the true proportion of those using AMFm-ACTs within 5% precision and assuming a 50% prevalence of utilization. Four research assistants with Ordinary National Diploma (OND) were trained for two days to assist in data collection. Research assistants were given packets of common antimalarial drugs including that of AMFm-ACTs (also known as antimalarial packet with the green leaf symbol) to show caregivers how to ascertain use of AMFm-ACTs. Data were collected over a period of one month.

The article "Awareness and Utilization of Affordable Medicine Facility-Malaria among Caregivers of Under-Five Children in Ibadan North-West Local Government Area, Oyo State" was published in 2013. Journal: Malar Res Treat.

#### 2.2.3. Sampling Technique

A cluster sampling of five enumeration areas was done. Based on the information from National Population Commission, Ibadan North-West has 509 enumeration areas [8]. It was estimated that an enumeration area consists of at least five hundred people and women in reproductive age group represent 22 percent of the total population. A total of 110 women were estimated to be found in each enumeration area. From the list of the enumeration areas 5 enumeration areas were randomly selected using table of random numbers. One household was randomly selected by balloting in all the clusters. This household served as the starting point and following a predetermined direction, women of reproductive age in consecutive households in each of the cluster were studied till the allocated sample size of 110 was achieved.

### 2.3. Data Collection

Participants were interviewed using a pretested semistructured questionnaire. Questionnaire was adapted from ACT watch household survey questionnaires used in seven African countries [9] and questions from the literatures that assessed the utilization of Artemisinin-Based Combination Therapy were also added. Questionnaire administration commenced after obtaining approval to conduct the study from Oyo state Ethical Review Committee and after informed consent was obtained from respondents. Information was collected on sociodemographic characteristics, knowledge on symptoms of malaria, treatment seeking for malaria, awareness of AMFm programme, utilization of AMFm-ACTs, and factors influencing utilization of AMFm-ACTs.

### 2.4. Data Analysis

Data were entered, cleaned, and analyzed using Statistical Package for Social Sciences version 15 software [10]. Frequencies, proportions, means, and standard deviations were used to summarize variables. The Chi-square test was used to determine associations between outcome and categorical explanatory variables. Logistic regression analysis was used to determine the predictors of using AMFm-ACTs. The level of statistical significance was set at 0.05. Use of AMFm-ACTs was defined as use of AMFm-ACTs within 24–48 hours of onset of fever. Information on awareness of AMFm-ACTs was ascertained by asking if the caregivers have heard about AMFm programme, if they have seen the packet of antimalarial drug with the green leaf symbol, sources where AMFm-ACTs was seen or heard, and if they knew what the symbol on the AMFm-ACTs packet meant. Concerning the meaning of the symbol on the drug packet, eight questions were asked and the maximum score that the respondents could get in this domain was 8. Respondents who scored above the mean were taken to have good knowledge and others having scores below the mean were taken to have poor knowledge. Factors influencing use of AMFm-ACTs were considered sociodemographic characteristics, socioeconomic status, awareness of AMFm-ACTs, Access to AMFm-ACTs, and knowledge on symptoms of malaria. Access was defined in terms of geographical accessibility to drug shops where AMFm-ACTs were being sold and also availability of AMFm-ACTs. Geographical access was considered good if it takes 30 minutes or less (irrespective of mode of transportation) for someone to reach the source of the drug. Socioeconomic status was calculated using the average monthly income of respondents. Respondents were thereafter classified into low and high socioeconomic class using $2 per day as a cut-off. People of low socioeconomic status were defined as people living below $2 per day [11, 12]. Respondents were categorized as having good knowledge on symptoms of malaria if they have scores above the mean scores, with the total obtainable score based on the number of questions asked and score of the response being 10 marks.

The article "Awareness and Utilization of Affordable Medicine Facility-Malaria among Caregivers of Under-Five Children in Ibadan North-West Local Government Area, Oyo State" was published in 2013. Journal: Malar Res Treat.

## 3. Results 

Four hundred seventy-eight caregivers participated in the study and their characteristics are shown in Table 1. The mean age of the respondents was 31.0 ± 5.4 years. Many of the caregivers 287 (60.3%) were between 25 and 34 years, 427 (89.3%) were married, and 287 (60.6%) were Christians. More than half 293 (61.7%) of the respondents had secondary education while 267 (55.9%) were traders and less than half 141 (32.2%) were of high socioeconomic status.

### 3.1. Knowledge on Symptoms of Malaria

Majority of the caregivers 415 (87.6%) had good knowledge of the symptoms of malaria in under-five children. Symptoms mentioned were fever 456 (95.6%), poor appetite 236 (49.5%), vomiting 132 (27.6%), and headache 83 (17.4%).

### 3.2. Awareness of Antimalarials and Treatment Pattern

Chloroquine was the most known antimalarial drug 465 (97.3%) and 312 (65.3%) knew about ACTs. ACTs was mentioned by 203 (42.5%) as the most effective antimalarial. This was followed by chloroquine 142 (29.7%), sulphadoxine-pyrimethamine 103 (21.5%), amodiaquine 19 (4.0%), and Quinine 6 (1.3%). One hundred seventy-three (36.2%) knew that ACT was the antimalarial drug recommended by the government for the treatment of malaria.

Most of the respondents 420 (88.8%) gave their febrile child antimalarial drug, 27 (5.6%) gave herbs, and 17 (3.6%) considered the fever not serious enough for the child to be given antimalarial drug. Out of those that gave their child antimalarial drug, 332 (79.2%) did so within 24 hours of onset of fever while 86 (20.6%) responded within 48 hours of onset of fever.

The article "Awareness and Utilization of Affordable Medicine Facility-Malaria among Caregivers of Under-Five Children in Ibadan North-West Local Government Area, Oyo State" was published in 2013. Journal: Malar Res Treat.

### 3.3. Awareness on AMFm

Respondents who were aware of AMFm programme were 43 (9.1%) and less than half 204 (42.9%) have seen the antimalarial packet that has the symbol of the Affordable Medicine Facility-malaria. Those who were aware of the programme got the information from diverse sources and the commonest source of information was through the radio 13 (31.7%). For those who have seen the antimalarial packet that has the AMFm symbol, the commonest place where they saw it was at the pharmacy 125 (62.8%). Out of those who have seen the symbol, only 97 (47.5%) had a good knowledge of what the symbol meant. Most of the respondents who mentioned they have seen the AMFm symbol 183 (89.7%) when shown the packet felt it meant nothing, 23 (11.3%) knew it meant subsidized antimalarial drug, and 17 (8.3%) knew it meant ACT.

### 3.4. Use of AMFm-ACTs

Overall, 123 (29.2%) used AMFm-ACT as their first line antimalarial drug (Table 2). The mean price of the drug was *₦*  242.0 ± 90.39 which is equivalent to $1.5 (±0.6). Forty-eight (39.7%) bought it from PPMVs which constituted the commonest source of AMFm-ACTs. About 43 (35%) mentioned that health workers prescribed AMFm-ACTs, 63 (51.2%) administered the drug based on self-medication, and 17 (13.8%) did so based on recommendation by neighbours, friends, and relations. More than half 67 (54.5%) cited effectiveness of the drug as the main reason for choosing it while 42 (34.1%) mentioned recommendation by people as a basis for buying the drug. Majority of the respondents 101 (82.1%) reported availability of the antimalarial whenever they go to buy. With regard to geographical access, 93 (89.4%) had good access to the drugs.

### 3.5. Factors Influencing AMFm-ACTs Drug Use

Factors influencing AMFm-ACTs use were determined using Chi-square test. Significant factors at 5% level of significance were put in the logistic regression model. Age group (25–34 years) (*P* < 0.05), public servants (*P* < 0.001), respondents with tertiary education (*P* < 0.001), respondents with high socioeconomic status (*P* < 0.001), respondents with poor knowledge of symptoms of malaria in under-five children (*P* < 0.05), awareness of AMFm-ACTs (*P* < 0.001), availability of AMFm-ACTs (*P* < 0.001), and sources of drug being private clinic (*P* < 0.001) were significantly associated with the use of AMFm-ACTs. On logistic regression only people who were aware of AMFm-ACTs predicted its use (AOR: 0.073; CI: 0.032–0.166) (Table 3).

## 4. Discussion

The success of Malaria Control Programme hinges on people's awareness of its existence and utilization of interventions provided. Many studies on AMFm have examined the affordability and availability of the drug from the providers' point of view. This study focused basically on the consumers/end users to see if they are aware, if they use the drug and factors influencing their use of the drug. Findings from this study showed that a high proportion of caregivers of children less than five were not aware of the initiative among caregivers of children less than five years. This finding was consistent with a study done in Jos which found that majority of the caregivers were not aware of Artemisinin-Based Combination Therapy when it was adopted as the treatment of first choice for uncomplicated malaria [13]. The commonest source of information on AMFm-Acts was the radio. A literature on knowledge, attitudes, and practices about malaria treatment and prevention in Uganda also found radio as the commonest source of information on malaria [14]. The mean price of AMFm-ACTs was $1.5 (±0.6). This price is more than the stipulated price for children's dose. Studies have shown that the price at which AMFm-ACTs are sold in some countries that has adopted the initiative was less than the unsubsidized ACTs but more than the government recommended retail price [3, 15]. For example, a study done in Nigeria and Ghana found the adult dose of AMFm-ACTs to be cheaper than non-AMFm drugs but more than the anticipated price by government [15]. This suggests that the objective of AMFm to increase affordability of the drug has been partly achieved. Although prices are much lower for AMFm-ACTs, research should still be carried out to explore why the drugs are being sold at prices higher than the stipulated government price by drug sellers and other healthcare providers.

The article "Awareness and Utilization of Affordable Medicine Facility-Malaria among Caregivers of Under-Five Children in Ibadan North-West Local Government Area, Oyo State" was published in 2013. Journal: Malar Res Treat.

An assessment of the use of antimalarial drugs 24–48 hours of onset of fever gave intriguing result. The study showed that a similar proportion of caregivers used chloroquine and AMFm-ACTs as their first line drugs. This is contrary to findings from nationally representative outlet surveys in six sub-Saharan countries in 2011 (Benin, the Democratic Republic of Congo, Madagascar, Nigeria, Uganda, and Zambia) which found that nonartemisinin monotherapies were the most commonly acquired antimalarial drugs for children less than five years of age. The result for Nigeria showed that chloroquine was mostly used [16]. Utilization of chloroquine has been fuelled by its comparatively low price, familiarity of these older products, past successful treatment experiences, and excessive pill burden of artemether-lumefantrine. However, use of AMFm-ACTs can be increased by scaling-up awareness campaign at community level by the government and, non-government organizations involved. There is a possibility of AMFm-ACTs knocking out cheap and long used antimalarials if this is done. This possibility is assumed based on the success of subsidized ACTs that were introduced in Kenya and Uganda [17]. Increased sensitisation about the treatment failure rates and the additional costs that could be incurred due to treatment failure both among health professionals and the community could also help to increase utilization of subsidised ACTs and caregivers desist from using chloroquine and SP [18].

Majority of the caregivers in this study got their drugs from PPMVs. The literature on treatment seeking pattern in sub-Saharan including Nigeria revealed that medicine sellers are widely used as sources of drug for malaria and fever [19, 20]. Majority of the caregivers reported availability of the drug whenever they go to buy it. This finding is in consonance with a study done in seven African countries in 2012 (Ghana, Kenya, Madagascar, Niger, Nigeria, Uganda, and Tanzania) which found out that there was increase in availability and market share of quality assured ACTs (QAACT) at the PPMVs except for Niger and Madagascar [3]. Another study carried out to determine Artemisinin-Based Combination Therapy availability and use in the private sector of five AMFm phase 1 countries found that market penetration of one or more AMFm QAACT was high both in rural and urban areas [21].

In this study only awareness predicted the use of AMFm-ACTs. This was similar to a study on insecticides treated net where awareness predicted the ownership and use of the nets [22]. Similarly, in a study in Kenya, community awareness activities were reported to have been instrumental to a substantial increase in ACT availability and coverage [23].

The main limitation of this study was that caregiver's pattern of use of AMFm-ACTs was estimated using caregiver's self-report. Recall bias may likely occur from this, but it was minimized by asking for their pattern of use in the last two weeks prior to the survey.

## 5. Conclusions

Findings from this study revealed that awareness of AMFm-ACTs was low and this translated to low utilization of AMFm-ACTs. This may hinder achieving the objectives of AMFm which are to expand access to ACTs. Scaling-up of programmes to increase awareness is needed to increase coverage.

## Figures and Tables

**Table 1:** Sociodemographic characteristics of the respondents.

Variable	Frequency	Percentage (%)
Age (yrs) *N* = 476		
15–24	58	12.2
25–34	287	60.3
≥35	131	27.5
Income *N* = 438		
Low socioeconomic status	297	67.8
High socioeconomic status	141	32.2
Level of education *N* = 475		
None	18	3.8
Primary	107	22.5
Secondary	293	61.7
Postsecondary	57	12.0
Marital status		
Married	427	89.3
Separated	1	1.3
Divorced	6	0.2
Single	38	7.9
Cohabiting	6	1.3
Occupation *N* = 478		
Trader	267	55.9
Artisans	128	26.8
Civil servant	55	11.5
Others*	28	5.9
Religion *N* = 472		
Christian	286	60.6
Islam	186	39.4

*Others were housewife, students, and auxiliary nurse.

The article "Awareness and Utilization of Affordable Medicine Facility-Malaria among Caregivers of Under-Five Children in Ibadan North-West Local Government Area, Oyo State" was published in 2013. Journal: Malar Res Treat.

**Table 2:** Use of Antimalarial drugs.

Antimalarial drugs used	Frequency	Percent (%)
Artesunate/amodiaquine	4	1.0
Artesunate	5	1.2
Amodiaquine	19	4.5
Artemether/lumefantrine	35	8.3
Sulphadoxine-pyrimethamine	112	26.6
Chloroquine	123	29.2
AMFm-ACTs	123	29.2

Total	421	100

**Table 3:** Logistic regression on predictors of use of AMFm-ACTs.

Variable	OR	95% CI lower	95% CI upper	*P* value
Occupation				
Trader (Ref.)	1.000			
Artisan	1.778	0.892	3.544	0.102
Civil servant	1.861	0.321	2.312	0.767
Others	1.273	0.324	4.999	0.730
Source of drug				
Supermarket (Ref.)	1.000			
Public facility	2.094	0.223	19.653	0.518
Private clinic	5.038	0.579	43.826	0.143
Pharmacy	1.547	0.225	10.644	0.657
PPMV	0.505	0.077	3.325	0.478
Level of education				
None (Ref.)	1.000			
Primary	0.386	0.053	2.802	0.347
Secondary	0.844	0.134	5.338	0.857
Postsecondary	1.502	0.201	11.215	0.692
Knowledge of symbol meaning				
Poor	1.178	0.530	2.616	0.688
Good (Ref.)	1.000			
Income				
Low socioeconomic status	0.527	0.266	1.043	0.066
High socioeconomic status (Ref.)	1.000			
Awareness of AMFm-ACTs				
No	0.073	0.032	0.166	0.000*
Yes (Ref.)	1.000			
Knowledge on symptoms malaria				
Good (Ref.)	1.000			
Poor	1.817	0.734	4.498	0.196
